This article has been retracted.

# Indomethacin-based stimuli-responsive micelles combined with paclitaxel to overcome multidrug resistance

**DOI:** 10.18632/oncotarget.22781

**Published:** 2017-11-30

**Authors:** Shuanghu Wang, Xueying Tan, Shujuan Li, Yunfang Zhou, Peiwu Geng, Ailian Hua, Aiping Deng, Zhihong Yu

**Affiliations:** ^1^ The Laboratory of Clinical Pharmacy, The Sixth Affiliated Hospital of Wenzhou Medical University, The People's Hospital of Lishui, Lishui 323000, China; ^2^ College of Pharmacy, Zhejiang Pharmaceutical College, Ningbo 315000, China; ^3^ Department of Pharmacy, The Central Hospital of Wuhan, Tongji Medical College, Huazhong University of Science and Technology, Wuhan 430000, China

**Keywords:** breast cancer, multidrug resistance, paclitaxel, indomethacin, drug delivery system

## Abstract

Development of multidrug resistance against antitumor agents is a major limiting factor for the successful chemotherapy. Currently, both amphiphilic polymeric micelles and chemosensitizers have been proposed to overcome MDR during chemotherapy. Herein, the redox-responsive polymeric micelles composed of dextran and indomethacin (as chemosensitizer) using a disulfide bond as the linker are prepared (DEX-SS-IND) for delivery of antitumor agent paclitaxel (PTX). The high level of glutathione in tumor cells selectively breaks the disulfide bond, leading to the rapid breakdown and deformation of redox-responsive polymeric micelles. The data show that DEX-SS-IND can spontaneously form the stable micelles with high loading content (9.48 ± 0.41%), a favorable size of 45 nm with a narrow polydispersity (0.157), good stability, and glutathione-triggered drug release behavior due to the rapid breakdown of disulfide bond between DEX and IND. *In vitro* antitumor assay shows DEX-SS-IND/PTX micelles effectively inhibit the proliferation of PTX-resistant breast cancer (MCF-7/PTX) cells. More impressively, DEX-SS-IND/PTX micelles possess the improved plasma pharmacokinetics, enhanced antitumor efficacy on tumor growth in the xenograft models of MCF-7/PTX cells, and better *in vivo* safety. Overall, DEX-SS-IND/PTX micelles display a great potential for cancer treatment, especially for multidrug resistance tumors.

## INTRODUCTION

Multidrug resistance (MDR) is well known as a crucial limiting factor for the successful chemotherapy [1]. Overexpression of multidrug resistance-associated proteins (MRPs) play a vital role in mediating efflux of chemotherapeutic agents from cells [2, 3]. To improve therapeutic outcomes, several strategies have been designed to suppress or reduce the activity of MRPs on the tumor cells. One effective strategy is to take advantage of MDR inhibitor or regulator, which can effectively reduce, and even reverse MDR via blocking the efflux of antitumor agents from tumor cells, and then increase intracellular drug concentration and improve therapeutic outcomes [4–7].

Paclitaxel (PTX) is extensively used as a chemotherapy medication in clinical practice, such as breast cancer, lung cancer, Kaposi sarcoma and cervical cancer [8]. However, MDR developed by tumor cells launch a challenge for oncotherapy during alone or combination with other antitumor drugs. So far, only three formulations of PTX are available in the market, namely Taxol^®^, Abraxane^®^ and Genexol^®^-PM. Taxol^®^ contains dehydrated alcohol and Cremophor EL, but the latter potentially causes hypersensitivity and nephrotoxicity [9]. To avoid side effects induced by Cremophor EL and enhance the antitumor activity, various materials have been used to develop new formulations. Abraxane, protein-bound PTX, is approved for breast cancer, lung cancer and pancreatic cancer [10], but it is too expensive to afford it. Moreover, no evidence indicates that Abraxane can be against MDR cancer. Similarly, Genexol®-PM, a PTX-loaded polymeric micelle, shows the good antitumor activity and tolerability, but there is also no evidence that it can suppress or reverse MDR. Therefore, it is desiderated to develop a new drug delivery system (DDS) to co-deliver PTX and MDR inhibitor to overcome MDR during oncotherapy.

Polymeric micelles effectively deliver hydrophobic antitumor agents benefiting from their unique advantages, especially for stimuli-responsive micelles that spontaneously form nanosized particles in aqueous medium and conditionally release the encapsulated drugs under the effects of external stimuli [11–13]. The micellar hydrophobic inner core can load water-insoluable agent, and hydrophilic outer shell is able to stabilize micelles and reduce potential recognition by the reticuloendothelial system (RES). Redox-responsive DDS is a reasonable strategy due to the intracellular higher glutathione (GSH) concentration than that in the extracellular environment. It was previously demonstrated that redox-responsive DDS kept stability in the circulation with low GSH level, but rapidly broke and released the encapsulated drugs under the effects of GSH [14].

In this study, redox-responsive micelles were prepared using dextran (DEX) as hydrophilic outer shell and indomethacin (IND) as hydrophobic inner core. Previous study showed IND inhibited MDR pump via regulating multi-drug resistance protein 1 (MRP1) promoter activity [15]. The obtained amphipathic polymer spontaneously formed micelles and effectively loaded hydrophobic PTX. The intracellular PTX release behaviors and antitumor activities of redox-responsive dextran-SS-indomethacin/paclitaxel (DEX-SS-IND/PTX) micelles were systematically assessed in this study.

## RESULTS AND DISCUSSION

### Synthesis and characterization of DEX-SS-IND

DEX-cystamine (DEX-SS, yield: 39.4%) was firstly synthesized by amide reaction in the presence of dicyclohexylcarbodiimide (DCC) and N-hydroxysuccinimide (NHS). Then, IND was conjugated to DEX-SS under the action of DCC and NHS to finally obtain DEX-SS-IND (yield: 35.8%) (Figure 1A). The synthetic route was provided in Supplementary Figure 1. The obtained DEX-SS-IND was confirmed using ^*1*^*H* nuclear magnetic resonance (^*1*^*H* NMR, Bruker AV-500spectrometer, Switzerland) and dimethylsulfoxide-*d*_6_used as a solvent. Figure 1B showed the ^*1*^*H* NMR spectra of DEX, IND and DEX-SS-IND. The characteristic peaks of DEX-SS-IND at 3∼4 ppm and 7∼8 ppm (c, d) belonged to DEX (a, -CH-) and IND (b, -CH-), suggesting DEX-SS-IND was conjugated successfully. In addition, insensitive micelle, DEX-IND, was used as a control, and its synthetic route and structure confirmation were provided in Supplementary Figure 2. The release profile of IND from DEX-SS-IND was also investigated and the result was shown in Supplementary Figure 3.

**Figure 1:** Preparation and characterization of DEX-SS-IND/PTX micelles **(A)** Schematic formation of DEX-SS-IND/PTX micelles. **(B)** ^*1*^*H* NMR spectra of dextran, indomethacin and DEX-SS-IND (a and c, -CH-, at 3∼4 ppm; b and d, -CH-, 7∼8 ppm) **(C)** Negative-stain transmission electron microscopy of DEX-SS-IND blank micelles and DEX-SS-IND/PTX micelles. Scale bar = 100 nm.

The obtained DEX-SS-IND possessed amphipathic characteristic that spontaneously formed micelles in aqueous medium. The aggregation behavior of DEX-SS-IND was investigated via measuring critical micelle concentration (CMC) using pyrene as a probe, and the CMC value was 31.6 μg/mL.

### Characterization and stability of DEX-SS-IND/PTX micelles

DEX-SS-IND/PTX micelles were prepared via solvent diffusion method, and characterized for by dynamic light scattering (DLS, Zetasizer 5000, UK) and transmission electron microscopy (TEM, Hitachi-7700, Japan). Table 1 summarized the micellar size, polydispersity index (PDI), drug loading (DL%) and encapsulating efficiency (EE%). The micellar size with PTX feeding ranging from 0 to 15% was less than that of blank DEX-SS-IND micelles, which was associated with the hydrophobic interaction between IND and PTX becoming stronger. Then, the increased micellar size was achieved with further enhanced drug feeding ratio.

**Table 1:** Characteristics of DEX-SS-IND/PTX micelles (n=3)

Feeding ratio(%)	Size (nm)	PDI	EE(%)	DL(%)
0 %	55.4 ± 6.3	0.206 ± 0.075	-	-
5 %	52.6 ± 5.8	0.185 ± 0.065	80.25 ± 4.3	4.27 ± 0.59
10 %	48.4 ± 5.3	0.169 ± 0.089	82.35 ± 5.8	6.45 ± 0.48
15 %	45.7 ± 4.3	0.157 ± 0.055	88.26 ± 4.8	9.48 ± 0.41
20 %	115.7 ± 8.6	0.228 ± 0.102	87.26 ± 6.3	12.6 ± 0.59

PDI, polydispersity index; EE(%), encapsulation efficiency; DL(%), drug loading; Feeding ratio(%).

Figure 1C showed the TEM images of blank DEX-SS-IND micelles and DEX-SS-IND/PTX micelles with 15% drug feeding, verifying their uniform spherical shape. The micellar size shown in the TEM images was smaller than that measured via DLS, the discrepancy of which was associated with the fact that DLS detected the hydrodynamic micelle size while TEM captured the dried state. DEX-SS-IND/PTX micelles with 15% drug feeding were used in the subsequent experiments.

The mean size and PDI of DEX-SS-IND/PTX micelles were monitored at different periods of time to assess the *in vitro* stability of micelles. As shown in Figure 2A and 2B, the size and PDI of DEX-SS-IND/PTX micelles had a little change after two weeks storage at 4°C, suggesting the colloidal stability of DEX-SS-IND/PTX micelles could be maintained at 4°C.

**Figure 2:** *In vitro* release behaviors and stability of DEX-SS-IND/PTX micelles **(A)** and **(B)** *In vitro* stability of DEX-SS-IND/PTX micelles at 4°C, including size and PDI. **(C)** The size changes of DEX-SS-IND/PTX micelles in the different reduction environments. ^*^ *P* < 0.05. **(D)** PTX release of DEX-IND/PTX and DEX-SS-IND/PTX micelles in PBS 7.4 with or without 10 mM GSH. **(E)** PTX release of DEX-SS-IND/PTX micelles in PBS 7.4 with various concentrations of GSH. **(F)** and **(G)** NR fluorescent images and quantification of DEX-SS-IND/NR or DEX-IND/NR micelles after incubation with different concentrations of GSH for 10, 20 and 40 min.

### Reduction responsive behaviors triggered by GSH

It was previously reported that the intracellular GSH concentration was approximately 0.5-10 mM, which was higher than that in the extracellular environment (ca. 2-20 μM) [14, 16]. Therefore, it was possible that the disulfide bond in DEX-SS-IND micelles could be rapidly reductive degraded in tumor cells. Therefore, *in vitro* reduction responsive behaviors of DEX-SS-IND micelles were investigated in pH 7.4 PBS with various GSH concentrations (0 μM, 10 μM, 2 mM, and 10 mM). Figure 2C showed micellar size changes responding to the various GSH concentrations. No obvious size changes after incubation with 10 μM GSH, suggesting the intact micellar structure. Namely, the integrity of DEX-SS-IND/PTX micelles could be maintained under such a GSH concentration similar with the GSH level in blood. Micellar size increased after incubated with 2 mM GSH, and significant enhanced size was observed under the condition of 10 mM GSH (both ^*^P < 0.05). Some aggregates emerged in DEX-SS-IND micelle solution after incubation with 10 mM GSH, implying the cleavage of redox-responsive disulfide bonds in the simulative reducing environment of tumor cells.

### GSH-triggered drug release

The *in vitro* redox-responsive release behaviors of DEX-SS-IND/PTX micelles were investigated in pH 7.4 PBS with various GSH concentrations (0 μM, 10 μM, 2 mM, and 10 mM). As shown in Figure 2D, no significant difference of PTX release behavior was observed in PBS with 0 μM and 10 μM GSH, the latter of which was similar to the mildly oxidizing in the extracellular environment (about 2-20 μM). In contrast, the accelerated PTX release was achieved in PBS with 2 mM and 10 mM GSH, indicating the enhanced GSH concentration led to the cleavage of disulfide bond and disassembly micellar structures. Figure 2E further demonstrated the accelerated PTX release behavior of DEX-SS-IND/PTX micelles compared with that of DEX-IND/PTX micelles was due to the redox-responsive cleavage of disulfide bonds in the high GSH environment.

The redox-responsive release behavior of DEX-SS-IND micelles was further confirmed via incubating Nile red-loaded DEX-SS-IND (DEX-SS-IND/NR) micelles in pH 7.4 PBS with various GSH concentrations (0 μM, 2 mM, and 10 mM). Free NR could be observed, but the encapsulated NR was unobservable due to the shielding effect [17]. The fluorescence intensity changes represented the NR release from micelles. As shown in Figure 2F and 2G, the NR release behavior of DEX-SS-IND/NR micelles showed time- and GSH concentration-dependence. In contrast, the changes of time and GSH concentrations had no effects on the NR release from DEX-IND/NR micelles.

### Intracellular drug release

The intracellular drug release behavior of redox-responsive DEX-SS-IND micelles against drug-resistant MCF-7/PTX cells were investigated using NR as fluorescent probe [17]. Buthionine sulfoximine (BSO) is a sulfoximine used to reduce the intracellular GSH concentration [18]. In this study, MCF-7/PTX cells and BSO-pretreated MCF-7/PTX cells were used as cell models with high GSH level and lower GSH level, respectively. The GSH level in MCF-7/PTX cells with and without BSO-pretreatment were measured using a GSH determination kit according to the manufacturer’s protocol. The results showed the GSH concentration in BSO-pretreated cells was reduced by approximately 60% (Figure 3A, ^*^P < 0.05).

**Figure 3:** **(A)** Intracellular GSH levels of MCF-7/PTX cells and BSO-pretreated MCF-7/PTX cells, ^*^ *P* < 0.05. **(B)** *In vitro* GSH-triggered NR release from DEX-IND/NR micelles and DEX-SS-IND/NR micelles (red) in MCF-7/PTX and BSO-pretreated MCF-7/PTX cells, Scale bar = 25 nm. **(C)** The semi-quantitative values of fluorescence intensity of (B). **(D)** Quantitative determination of GSH-triggered NR release via flow cytometry. **(E)** The intracellular concentration of PTX in the DEX-SS-IND/PTX micelles at different time points (6 and 24 h). Data were presented as mean ± SD (n = 3), ^*^ *P* < 0.05. **(F)** Representative western blot analysis of MRP1 in MCF-7/PTX cells treated with DEX-SS-IND,β-actin was used as control. **(G)** Densitometric analysis for detecting thelevels of MRP1. Values were normalized against β-actin. Data were presented as mean ± SD (*n* = 3), ^*^P < 0.05.

5 × 10^4^ cells/well of MCF-7/PTX cells were cultured in a 24-well plate and kept at 37°C for 24 h. Then, DEX-IND/NR and DEX-SS-IND/NR micelles were added and further incubated for 1, 5 and 10 h, respectively. The intracellular NR release behaviors were visualized using laser scanning confocal microscope (CLSM, Olympus, Japan). We found that the NR fluorescence signal in MCF-7/PTX cells treated with DEX-SS-IND/NR micelles showed time-dependence. In contrast, the NR fluorescence signal was lower in cells treated with DEX-IND/NR micelles, suggesting NR could be released from redox-responsive DEX-SS-IND/NR micelles triggered by intracellular high GSH concentration while DEX-IND/NR micelles were independent from reducing tumor intracellular space. Moreover, only a few red fluorescent signals were observed in BSO-pretreated cells, further demonstrating the redox-responsive activity of DEX-SS-IND/NR micelles. Flow cytometry was also used and the results (Figure 3D) were in accordance with CLSM results.

### Cellular uptake studies

Internalization of DEX-SS-IND/PTX micelles by MCF-7 and MCF-7/PTX cells was quantitatively investigated via determining intracellular PTX concentration by HPLC method [19]. 5 × 10^4^ cells/well of cells were cultured in a 24-well plate and kept at 37°C for 24 h. Then, PTX, PTX + IND, DEX-IND/PTX, and DEX-SS-IND/PTX micelles were added and incubated for 6 and 24 h, respectively. After that, the cells were harvested and lysed with RIPA buffer to release the intracellular PTX for HPLC determination. Intracellular PTX content was expressed as the amount (nmol) of PTX associated with a unit weight (1 mg) of cellular protein. Protein contents of cell lysate were measured using BCA protein assay reagent kit [19].

As shown in Figure 3E, the internalization by MCF-7 cells showed the time-dependence. The intracellular PTX contents in cells incubated with DEX-IND/PTX and DEX-SS-IND/PTX micelles were significantly higher than those incubated with PTX and PTX + IND, which was due to the enhanced cellular uptake with micelles in comparison to free drugs (both ^*^P < 0.05). Compared with MCF-7 cells, the internalization of PTX by MCF-7/PTX cells was decreased remarkably under the effect of MRPs, while intracellular PTX contents were significantly enhanced with the help of IND. In addition, the intracellular PTX content in cells incubated with DEX-SS-IND/PTX micelles were significantly higher than incubated with DEX-IND/PTX micelles (^*^P < 0.05).

### MRP1 expression and activity assay

The reversal effect of DEX-SS-IND on drug transporters was investigating via western blot to assess the expression of MRP1 protein. As showed in Figure 3F and 3G, the expression of MRP1 in MCF-7/PTX cells was significantly higher than that in MCF-7 cells (^*^P < 0.05), whereas the MRP1 expressions were significantly reduced in MCF-7/PTX cells treated with DEX-SS-IND and IND (both ^*^P < 0.05). MRP1 plays a key role in MDR and is overexpressed MCF-7/PTX cells in comparison to MCF-7 cells. It protects cells from antitumor agents via pumping drugs out of the cells and reducing intracellular drug concentrations. As previous studies indicated, IND could overcome MDR via reducing the export functions of MRP1 [20]. We demonstrated the reversal effect of DEX-SS-IND on the expression of MRP1 in MCF-7/PTX cells in this study.

### *In vitro* antitumor activity

MTT assay was used to assess cytotoxicity of DEX-SS-IND in MCF-7 and MCF-7/PTX cells, and the results (Figure 5A and 5B) showed the cell viability after 48 h incubation with various concentration levels ranging from 1-400 μg/mL, suggesting negligible toxicity against MCF-7 and MCF-7/PTX cells.

**Figure 4:** *In vitro* anti-tumor activity of DEX-SS-IND/PTX micelles **(A)** and **(B)** MTT assay of blank DEX-SS-IND and DEX-IND micelles against MCF-7 and MCF-7/PTX cells after 48 h incubation (n = 3). **(C)** MTT assay of PTX-based formulations against MCF-7 and MCF-7/PTX cells after 48 h incubation (n = 3), ^*^ *P* < 0.05. **(D)** and **(E)** Imaging and quantitative analysis of live (green) cell assay for exposure of MCF-7/PTX cells to different PTX-based formulations, Scale bar = 100 nm.

**Figure 5:** **(A)** Maximum tolerated dose of DEX-SS-IND/PTX (n = 3). **(B)** Plasma concentration-time curves after intravenous administration of Taxol, DEX-IND/PTX and DEX-SS-IND/PTX micelles (equivalent 10 mg/kg PTX). **(C)** Biodistribution in tissue in mice after intravenous administration of Taxol, DEX-IND/PTX and DEX-SS-IND/PTX micelles at equivalent 10 mg/kg PTX for different times (6 and 12 h). Data were presented as mean ± SD (*n* = 4), ^*^ *P* < 0.05.

Then, *in vitro* antitumor activity of DEX-SS-IND/PTX micelles was investigated in comparison to PTX, PTX + IND and redox-irresponsive DEX-IND/PTX micelles. As shown in Figure 5C, PTX-based formulation dose-dependently reduced the viability of MCF-7 cells. However, the *in vitro* antitumor activity of PTX against MCF-7/PTX cells was reduced significantly (^*^P < 0.05), which was due to the simple diffusion of PTX into MCF-7/PTX cells, but its accumulation and retention in MCF-7/PTX cells was significantly reduced under the effect of efflux activity of MRPs overexpressed on MCF-7/PTX cells. Compared with PTX, DEX-IND/PTX and DEX-SS-IND/PTX micelles had better antitumor activity against MCF-7/PTX cells, suggesting the internalization of micelles via endocytosis contributed to the increased PTX accumulation in MCF-7/PTX cells. In addition, the antitumor activity of PTX + IND was also better than PTX, suggesting the increased cytotoxicity of PTX by IND in MCF-7/PTX cells in comparison to PTX. Benefiting from chemosensitizer IND and redox-responsive DDS, DEX-SS-IND/PTX micelles showed the best antitumor activity in MCF-7/PTX cells. The enhanced antitumor activity of DEX-SS-IND/PTX micelles was also demonstrated by staining with Calcein AM, and DEX-SS-IND/PTX micelles led to the highest MCF-7/PTX cell death in comparison to other PTX-based formulations (Figure 4D and 4E).

### Maximum tolerated dose

The maximum tolerated dose (MTD) of DEX-SS-IND/PTX micelles was investigated in Balb/c nude mice bearing MCF-7/PTX tumors. Mice were respectively treated with Taxol, DEX-IND/PTX and DEX-SS-IND/PTX micelles, and body weight was monitored daily for two weeks. As shown in Figure 5A, more than 20% weight loss was observed in mice treated with 30 mg/kg Taxol. In contrast, the reduction in body weight was lower than 6% in mice treated with DEX-IND/PTX and DEX-SS-IND/PTX micelles at the same dose, suggesting micelle-based formulation could greatly enhance tolerance degree of PTX. Moreover, 50 mg/kg DEX-SS-IND/PTX micelles led to the weight loss of < 10%, whereas the same dose of DEX-IND/PTX micelles caused weight loss of > 10%. It was speculated that the MTD of DEX-SS-IND/PTX micelles was higher than that of DEX-IND/PTX micelles, which was associated with more PTX responsively released from DEX-SS-IND/PTX micelles at tumor sites and accordingly lesser PTX distributed in normal tissues.

### Pharmacokinetics and biodistribution

The mean plasma concentration-time curves of PTX in male Sprague-Dawley rats (200 ± 20 g) after a single intravenous administration of Taxol (10 mg/kg), DEX-IND/PTX (corresponding to 10 mg/kg PTX) or DEX-SS-IND/PTX (corresponding to 10 mg/kg PTX) micelles were determined with HPLC and shown in Figure 5B. Taxol was cleared quickly from the bloodstream at initial 6 h after intravenous administration, presenting a typical biphasic pattern including quick distribution phase (t_1/2α_ = 1.066± 0.335 h) and fast terminal elimination phase (t_1/2β_= 5.26 ± 1.843 h). In contrast, the reduction of plasma drug concentration in rats treated with DEX-IND/PTX or DEX-SS-IND/PTX micelles was significantly delayed (t_1/2α_ = 1.845 ± 0.09, t_1/2β_ = 9.756 ± 2.798; t_1/2α_= 2.049 ± 0.378, t_1/2β_ = 9.992 ± 2.371), respectively.

The mean pharmacokinetic parameters were calculated and summarized in Table 2. Compared with Taxol, the area under concentration curve (AUC_0-∞_) in DEX-IND/PTX and DEX-SS-IND/PTX micelles was significantly increased from 820.841 ± 95.36 μg/mL·h to 4364.078 ± 1715.462 μg/mL·h and 3575.572 ± 1507.981 μg/mL·h, respectively. The mean residence time (MRT) of DEX-IND/PTX (10.225 ± 1.561 h) and DEX-SS-IND/PTX (8.462 ± 2.586 h) micelles was 1.98- and 1.64-fold increase for free Taxol (5.143 ± 1.152 h), respectively. In addition, the apparent volume of distribution (V_d_) and clearance rate (CL) of DEX-SS-IND/PTX was significantly reduced in comparison to Taxol (^*^ *P* < 0.05), whereas no significant difference was observed between DEX-SS-IND/PTX and DEX-IND/PTX micelles. The obtained data demonstrated the increased systemic circulation time and high stability of DEX-SS-IND/PTX micelles to achieve efficient accumulation of PTX in tumor tissue and enhanced antitumor effects.

**Table 2:** Plasma pharmacokinetic parameters of DEX-SS-IND/PTX (10 mg/kg PTX) micelles

	PTX	DEX-IND/PTX	DEX-SS-IND/PTX
t_1/2α_/h	1.07 ± 0.34	1.85 ± 0.09	2.05 ± 0.38^*^
t_1/2β_/h	5.26 ± 1.84	9.76 ± 2.80	9.99 ± 2.37
MRT_0-∞_/h	5.14 ± 1.15	10.23 ± 1.56	8.46 ± 2.59
AUC_0-∞_/μg·mL^-1^·h^-1^	820.84 ± 95.36	4364.08 ± 1715.46	3575.57 ± 1507.98
C_max_/μg·mL^-1^	29.70 ± 2.66	52.40 ± 5.37	52.23 ± 3.60
CL/mL·h^-1^·kg^-1^	8.58 ± 1.47	2.19 ± 1.28	3.06 ± 1.29^*^
V_d_/mL·kg^-1^	67.47 ± 9.17	29.30 ± 4.20	28.40 ± 4.18^*^

t_1/2_, half-life; C_max_, peak concentration; AUC, area under the concentration-time curve; MRT, mean residence time; CL, clearance rate; V_d_, apparent volume of distribution.

To determine the accumulated PTX in tumors and normal tissues at 24 and 48 h after intravenous administration of PTX-based formulations at 10 mg/kg PTX equivalent, the tissue samples were processed according to the previous study by Liang et al. [21] and the results were shown in Figure 5C. After administration for 24 and 48 h, the accumulations of DEX-IND/PTX and DEX-SS-IND/PTX in tumors were significantly enhanced compared with Taxol. The increased accumulation was associated with the following two reasons: (1) the micellar hydrophilic outer shell protected PTX-loaded micelles from specific recognition by the reticuloendothelial system (RES) [22]. (2) the enhanced penetration and retention (EPR) effect led to the increased accumulation of PTX in tumors [23]. In addition, the accumulation of PTX released from DEX-SS-IND/PTX in tumor was higher than that released from DEX-IND/PTX, which could be attributed to the redox-responsive release behavior of DEX-SS-IND/PTX micelles due to the reducing intracellular environment. In contrast, the accumulation of PTX released from DEX-IND/PTX and DEX-SS-IND/PTX in normal tissues was significantly reduced in comparison to Taxol, which indicated that micelles could ameliorate PTX-induced toxicity to normal tissues.

### *In vivo* antitumor efficacy and histological analysis

*In vivo* antitumor efficacy of DEX-SS-IND/PTX micelles was investigated in Balb/c nude mice bearing MCF-7 and MCF-7/PTX tumors. The nude mice began to receive PTX-based formulations when tumor volumes were approximately 100 mm^3^, and treated with (1) Saline, (2) DEX-SS-IND, (3) Taxol (10 mg/kg), (4) DEX-IND/PTX (PTX 10 mg/kg) micelles and (5) DEX-SS-IND/PTX (PTX 10 mg/kg) micelles once every 2 days on days 0, 2, 4, 6 and 8 (the initial administration was set as day 0).

As shown in Figure 6A, Taxol, DEX-IND/PTX and DEX-SS-IND/PTX micelles all effectively inhibit the growth of MCF-7 tumors, and DEX-SS-IND/PTX micelles showed the best therapeutic outcomes (*vs* Taxol and DEX-IND/PTX). For MCF-7/PTX tumors, Taxol showed little inhibition of the tumor growth at the end of the treatment (*vs* Saline). DEX-IND/PTX micelles displayed moderate tumor inhibition, and DEX-SS-IND/PTX micelles showed the best antitumor outcomes verified by the significant difference in the tumor volume.

**Figure 6:** *In vivo* antitumor efficacy of DEX-SS-IND/PTX micelles **(A)** and **(B)** Tumor growth curves of mice after administrated with different PTX-based formulations (n = 6). **(C)** MCF-7/PTX xenograft tumor sections stained with H&E for the histological examination, with Ki67 for the tumor proliferation analyses and with TUNEL for the apoptosis analyses (200 ×).

Further histological analysis was used to assess the antitumor efficacy of DEX-SS-IND/PTX micelles on MCF-7/PTX tumors. The tumor sections were stained with hematoxylin and eosin (H&E), immunohistochemical staining Ki-67 and terminal deoxynucleotidyltransferase mediated UTP end labeling (TUNEL). As shown in first panel of Figure 6C, the tumor sections in the saline and DEX-SS-IND group both displayed intact nuclei morphology and uniform color. In contrast, the tumor sections in the drug-treated group showed darker color and wider intracellular spaces, even nuclei lysis, especially in DEX-SS-IND/PTX micelle group. Then, the TUNEL images were used to assess the apoptosis of DEX-SS-IND/PTX micelles (The second panel of Figure 6C). From these images, the dark brown represents apoptotic cells, accompanied with the condensed chromatin and cracked nuclear membrane [24]. The results were in accordance with the tumor growth curves, and DEX-SS-IND/PTX micelles showed the highest apoptotic activity in comparison to other treatment formulations. Lastly, anti-proliferation effect of DEX-SS-IND/PTX micelles was assessed via observing proliferating marker, Ki-67. DEX-SS-IND/PTX micelles effectively reduce cell proliferation compared with other PTX-based formulations. All these results provided the sufficient evidence that DEX-SS-IND/PTX micelles effectively overcame MDR tumors.

### Toxicity

Although Taxol could effectively inhibit the growth of MCF-7 xenograft tumors, the body weight of tumor-bearing mice inevitably reduced in comparison to saline group (Figure 7A), suggesting systemic toxicity was caused by Taxol at dose of 10 mg/kg. Taxol showed little therapeutic efficacy for the inhibition of MCF-7/PTX xenograft tumors at the above dosage, but it led to the significant reduction in body weight (Figure 7B). In contrast, the PTX-induced systemic toxicity was improved greatly in mice treated with DEX-SS-IND/PTX and DEX-IND/PTX micelles, suggesting PTX-loaded micelles led to the increased drug accumulation in tumor location and then reduced exposure of normal tissues.

**Figure 7:** Reduced systemic toxicity of PTX by DEX-SS-IND/PTX micelles **(A)** and **(B)** Body weight changes of nude mice bearing MCF-7 and MCF-7/PTX xenograft tumors, respectively (n = 6). **(C)** H&E staining microphotos of heart and liver tissues of mice bearing MCF-7/PTX xenograft tumors at the end of antitumor inhibition test (200×).

Further histological analysis was performed to assess the toxicity of PTX-based formulations because Taxol inevitably caused organ damages. As shown in Figure 7C, no pathological changes were observed in the heart and liver of mice receiving saline and DEX-SS-IND, but Taxol induced tissue damages. In contrast, DEX-SS-IND/PTX micelles significantly alleviated PTX-induced toxicity in non-target organs. Given micelles with size less than 100 nm are preferred for tumor targeting and redox-responsive PTX release behavior, DEX-SS-IND/PTX micelles might reduce PTX accumulation in normal tissues and ameliorate PTX-induced toxicity. All these data confirmed that DEX-SS-IND/PTX micelles significantly reduced PTX-induced toxicity.

## MATERIALS AND METHODS

### Synthesis and characterization of DEX-SS-IND

DEX-SS-IND was synthesized following a two-step process. Briefly, the reaction of DEX and cystamine (molar ratio, 1:10) dissolved in anhydrous DMSO was performed in the presence of DCC and NHS for 24 h at 50°C under the protection of nitrogen. After the reaction, the reaction solution was dialyzed against pure water for 48 h and then lyophilized to achieve DEX-SS. Then, DEX-SS-IND was synthesized via the reaction of DEX-SS and IND in the presence of DCC and NHS for 24 h at 50°C under the protection of nitrogen. The reaction solution was dialyzed against pure water, centrifugated at 15 000 rpm to get rid of water-insoluble byproducts and then lyophilized.

The obtained DEX-SS-IND was confirmed using ^*1*^*H* NMR spectroscopy (Bruker, Switzerland), and dimethylsulfoxide-*d*_6_ were used as solvent. The CMC value of DEX-SS-IND was measured using pyrene as the fluorescent probe [25].

### Preparation and characterization of DEX-SS-IND/PTX micelles

DEX-SS-IND/PTX micelles were prepared via the dialysis method [25]. Briefly, 10 mg DEX-SS-IND was dispersed in 5 mL pure water, and PTX was dissolved in ethanol of 2 mg/mL. Then, PTX ethanol solution was gradually added into DEX-SS-IND solution. After stirring for 30 min, the mixed solution was dialyzed and centrifuged to get rid of unencapsulated PTX [25].

The sizes and PDI were determined with DLS, and micellar morphology was examined using a Hitachi-7700 transmission electron microscopy (Hitachi, Tokyo, Japan). To assess the stability of micelles, their size and PDI were recorded after storage at 4°C for 2 weeks.

### Encapsulation efficiency and drug loading

The encapsulation efficiency (EE%) and drug loading (DL%) were determined as described previously [26]. Briefly, 0.5 mL DEX-SS-IND/PTX micelle solution was dissolved in 9.5 mL DMSO to dissolve all PTX. The concentration of PTX was determined using high performance liquid chromatography (HPLC) on an Agilent C18 (250 mm × 4.6 mm, 5 μm) column with a linear range from 1 to 20 μg/mL. Acetonitrile/water (45:55, v/v) was used as the mobile phase, and the detection wavelength was set as 240 nm with flow rate at 1.0 mL/min at 30°C [19]. The DL% and EE% of PTX were calculated as following formula:

DL% = (weight of PTX in micelles/Total weight of micelles) × 100%

EE% = (weight of PTX in micelles/Feeding amount of PTX) × 100%

### *In vitro* redox-responsive drug release

*In vitro* PTX release behavior of DEX-SS-IND/PTX micelles was investigated via the dialysis method [27]. Brifely, 2 mL DEX-SS-IND/PTX micelles were placed in dialysis bag (MWCO: 7.0 KDa) and suspended in 30 mL PBS solution with various GSH concentrations (0 μM, 10 μM, 2 mM, and 10 mM) and 2 M sodium salicylate. At designated times, 1 mL sample was collected and then exchanged with an equal volume of fresh media. The PTX concentration was measured via HPLC method.

Moreover, the micellar release behaviors triggered by GSH were investigated using fluorescence imaging. Briefly, NR was used as a model drug and its fluorescence intensity changes represented the degree of drug release [27]. Therefore, the release behavior of DEX-SS-IND/NR micelles could be evaluated via observing the fluorescence changes. DEX-SS-IND/NR or DEX-IND/NR micelles were exposure to pH 7.4 PBS with various GSH concentrations (0 μM, 2 mM, and 10 mM) for 10, 20 and 40 min, and fluorescence changes were observed using the *In vivo* Imaging System (DXS4000PRO, Kodak, USA)

### Cellular uptake of DEX-SS-IND/PTX micelles

For quantitative cellular uptake of PTX-loaded micelles, 5 × 10^4^ cell/well of MCF-7 and MCF-7/PTX cells were cultured in a in a 24-well plate and kept at 37°C for 24 h. Subsequently, PTX, PTX+IND, DEX-IND/PTX micelles and DEX-SS-IND/PTX micelles were added and further incubated for 6 and 24 h, respectively. RIPA buffer was used to release the intracellular PTX for HPLC analysis.

### Intracellular drug release

The intracellular drug release behaviors triggered by GSH were investigated using CLSM. The GSH levels in drug-resistant MCF-7/PTX cells and BSO-pretreated MCF-7/PTX cells were determined using a GSH determination kit. 5 × 10^4^ cell/well of MCF-7/PTX cells were cultured in a in a 24-well plate and kept at 37°C for 24 h. Subsequently, DEX-SS-IND/NR and DEX-IND/NR micelles were added into cells with or without BSO-pretreatment and further incubated for 1, 5 and 10 h, respectively. The intracellular NR release behaviors were visualized using CLSM. The intracellular NR fluorescence content was recorded using flow cytometry.

### Cytotoxicity assay

The cytotoxicity of DEX-SS-IND/PTX micelles against MCF-7 and MCF-7/PTX cells was assessed by MTT assay [28, 29]. 5 × 10^3^ cell/well of cells were cultured in a in a 24-well plate and kept at 37°C for 24 h. Subsequently, a series of concentrations of PTX-based formulation were added and further incubated for 48 h. Afterward, MTT solution (5.0 mg/mL) was added and kept for additional 4 h. The culture medium was replaced with 200 μL DMSO dissolve the purple formazan. Finally, the absorbance at 570 nm was determined using a micro plate reader, and viability was expressed as the percentage of the control. In addition, MCF-7/PTX cells pretreated with PTX-based formulation were stained with Calcein AM and observed using a fluorescence microscope.

### Western blot

Western blot was performed as previously described [30]. Primary antibodies for anti-MRP1 (1:2000, Abcom) and anti-β-actin (1:2000, proteintech) were used and protein bands were visualized using ECL Western Blotting Detection Kit (Beyotime Biotechnology, Shanghai, China). Band densitometry was calculated using Quantity One Software (Bio-Rad).

### Maximum tolerated dose

BALB/c mice bearing MCF-7/PTX tumors were treated with Taxol, DEX-IND/PTX and DEX-SS-IND/PTX micelles, respectively, and their body weight were monitored daily for 2 weeks. 10% weight change was determined to be part of significant clinical symptoms. 20% weight change was determined to attributable to lethal clinical signs [31].

### Pharmacokinetics

Healthy male SD rats (200 ± 20 g) were randomized to receive Taxol, DEX-IND/PTX and DEX-SS-IND/PTX micelles, respectively at PTX dose of 10 mg/kg body weight (n = 6). At designated times, blood samples were collected from orbit for HPLC analysis. The plasma samples (250 mL) were mixed with extract liquor (50 mL pH 5.0 sodium acetate buffer, 25 mL methanol and 6mL diethyl ether) and vortexed for 5 min. Then, the mixed liquor was centrifuged at 3 000 rpm for 10 min, and the supernatant was transferred to the tubes and evaporated to dryness under the nitrogen flow. The residual was redissolved in 200 μL methanol and centrifuged at 12 000 rpm for 10 min. 20 μL of supernatant was injected for HPLC determination. The PTX content in the plasma was determined by the HPLC assay described above.

### Biodistribution studies

Male BALB/c nude mice bearing MCF-7/PTX xenograft tumor cells were intravenously injected with various formulations at a dose of 10 mg/kg PTX (n = 4). At indicated times, mice were sacrificed by cervical dislocation and tissue samples were harvested and stored at -70°C until analyzed for PTX. The HPLC analysis for PTX was the same as mentioned above.

### *In vivo* anti-tumor activity

*In vivo* anti-tumor activity of DEX-SS-IND/PTX micelles was investigated in male BALB/c nude mice bearing MCF-7/PTX xenograft tumor cells. The nude mice began to receive various formulations when tumor volumes were approximately 100 mm^3^.

Group 1, Saline; Group 2, DEX-SS-IND; Group 3, Taxol (10 mg/kg); Group 4, DEX-IND/PTX (PTX 10 mg/kg) micelles; Group 5, DEX-SS-IND/PTX (PTX 10 mg/kg). The formulations were intravenously administrated once every 2 days on days 0, 2, 4, 6 and 8 (the initial administration was set as day 0) [25]. The tumor volume and body weight were monitored every 4 days and volume was calculated as the following formula [32]:

V_tumor_ (cm^3^) = ((breadth)^2^ × length)/2

### Histological examination

On day 36 after intravenous administration, mice were sacrificed, and organs (including heart and liver) and tumor were excised. The samples were immediately fixed in 4% formaldehyde solution and embedded in paraffin. The sections were stained with H&E. In addition, tumor section was stained with Ki-67 and TUNEL. The images were visualized using an optical microscopy (Olympus, Japan).

### Statistical analysis

The statistical significance of differences was analyzed via Student’s *t*-test, and mean differences with *P* < 0.05 were considered statistically significant. Pharmacokinetic data were analyzed using the Drug and Statistics Software (DAS 2.0). All data are expressed as the mean ± standard deviation of the independent measurements.

## CONCLUSION

In summary, the PTX-loaded micelles were prepared successfully based on DEX and IND, which could sensibilize the anti-tumor activity of PTX. The obtained DEX-SS-IND/PTX micelles showed the redox-responsive drug release behavior because the disulfide bond between DEX and IND was cleaved under reducing conditions, leading to the micellar disassembly and drug release. Intracellular PTX accumulation was significantly enhanced benefiting micellar endocytosis pathway and chemosensitizer IND that reduced MRPs-mediated PTX efflux. Both *in vitro* and *in vivo* assays demonstrated that DEX-SS-IND/PTX micelles could effectively inhibit the growth of MCF-7/PTX cells. Overall, the results indicated that DEX-SS-IND/PTX micelles showed great potential for overcoming drug-resistance during oncotherapy.

## SUPPLEMENTARY MATERIALS FIGURES


